# Early Detection and Management of Massive Intraoperative Pulmonary Embolism in a Patient Undergoing Repair of a Traumatic Acetabular Fracture

**DOI:** 10.1155/2018/7485789

**Published:** 2018-10-01

**Authors:** Tobechi E. Okoronkwo, XueWei Zhang, Jessica Dworet, Matthew Wecksell

**Affiliations:** New York Medical College-Westchester Medical Center, USA

## Abstract

A 73-year-old male with history of hyperlipidemia and osteoarthritis was transferred from an outside hospital after a fall from a ladder at home. He sustained a severe right sided acetabular fracture involving the femoral head, requiring operative repair. Preoperative evaluation was unremarkable except for oxygen saturation < 95 %. After induction of anesthesia and surgical positioning, the patient went into cardiac arrest. After intraoperative cardiopulmonary resuscitation (CPR) and placement on extracorporeal membrane oxygenation (ECMO), the patient stabilized. Cardiac catheterization revealed a large left pulmonary embolism. Here, we discuss the etiology and management of intraoperative pulmonary embolism.

## 1. Introduction

Perioperative pulmonary emboli (PE) in trauma patients are common. The incidence of thromboembolic events in trauma patients has been estimated at up to 63% [1] and the incidence of subclinical thromboemboli is higher still. The associated mortality of PE has reportedly been greater than 50% [2]. While timely diagnosis and treatment of PE can significantly improve patient survival [3], PE can be difficult to detect prior to hemodynamic collapse. Massive pulmonary embolism is often associated with physiologic instability characterized by acute right ventricular dysfunction, hypoxemia unresponsive to conventional therapy and cardiac arrest. Treatment of patients following massive PE with persistent shock includes installation of extracorporeal membrane oxygenation (ECMO), emergent pulmonary embolectomy, and thrombolysis. There lacks an overall consensus regarding which is the gold standard treatment modality [4].

While the American Society of Anesthesiologists (ASA) standard monitors have their role in diagnosis of PE, typically by demonstrating cardiovascular collapse, monitoring modalities like transesophageal echocardiography (TEE) and pulmonary artery catheters (PACs) have greater specificity and sensitivity. TEE and PACs can aid in therapeutic management of PE, especially in the hands of experienced personnel. While diagnostically helpful, TEE and PACs are not incorporated at the beginning of a standard orthopedic operation in a patient with no significant medical history. Here, we present a case of pulmonary embolism occurring after the induction of anesthesia and positioning in a patient with an extensive right acetabulum fracture. Our goal is to evaluate the available modalities for early detection and supportive care after hemodynamic collapse. The patient's family has given written consent to publish this case report.

## 2. Case Presentation

The patient is a 73-year-old male who was transferred from an outside hospital for repair of a right acetabulum fracture involving the femoral head after falling approximately 8-feet from a ladder while painting his house. Past medical history was significant for hyperlipidemia and osteoarthritis. Baseline metabolic equivalents were greater than four. Aside from a cataract extraction, the patient had no other operations. He denied any allergies. Prior to presentation, the patient was on Aspirin 81 mg daily for cardiovascular disease prevention and Atorvastatin 20 mg daily for hyperlipidemia. Computed tomography (CT) without contrast showed an acute, comminuted, and displaced fracture of the right acetabulum involving both posterior and anterior acetabular walls. The right femoral head was superiorly and laterally displaced with impaction fracture to its inferior and medial aspects. There were bone fragments within the right gluteus musculature, and the high attenuation in tissue density represented blood product within. Prior to surgery, the orthopedic team made an effort to reduce the patient's right acetabulum fracture with tibial traction pin under conscious sedation with midazolam, fentanyl, and ketamine in the emergency department. During the closed reduction, the patient experienced a brief period of respiratory depression. For approximately two minutes, his oxygen saturation was 85-86%, which improved to 95% with Narcan reversal. The emergency department record also noted that the patient had premature ventricular contractions on the electrocardiogram (EKG) at this time. After the closed reduction, the orthopedic team opted to monitor the patient on continuous telemetry for 24 hours and take the patient for open reduction and internal fixation of the right acetabulum the next day. He was not on prophylactic anticoagulation for this preoperative period.

Prior to entering the operating room, the patient's vital signs were stable: blood pressure 120/64, heart rate 73 beats per minute, respiratory rate 18 per minute, oxygen saturation 95%, and temperature 98.6 Fahrenheit. Neurological exam was significant for limited right knee flexion (<30 degrees). Otherwise, overall sensation was intact and right deep tendon reflex was intact. Hemoglobin was 11.6, down from 13.4 on admission. Coagulation tests showed elevated prothrombin time at 12.8, partial thromboplastin time 26.7, and international normalized ratio 1.20. In the OR, the patient was induced with standard dosing of midazolam, fentanyl, lidocaine, propofol, and succinylcholine. Phenylephrine was given preemptively on induction to avoid hypotension. Intubation was uncomplicated. Patient had two 20g peripheral intravenous catheter in place, and a left radial arterial line was placed after intubation. Despite premedication with phenylephrine, the patient became hypotensive with systolic blood pressure (SBP) in the 80s, median arterial pressure < 65. Boluses of ephedrine and phenylephrine were given, and a phenylephrine infusion was started thirty minutes after induction. The patient initially responded appropriately to treatment (SBP > 100). Due to concern for sciatic nerve injury, intraoperative somatosensory evoked potential (SSEP) monitoring was performed, and general anesthesia was maintained with propofol at 100 mcg/kg/min and remifentanil at 0.2 mcg/kg/min, in addition to 0.5% end tidal sevoflurane.

Upon patient positioning to the right lateral decubitus position from supine, the patient's SBP acutely declined into the 50s and the patient became hypoxic with an oxygen saturation of 88%. His hypotension was no longer responsive to phenylephrine or ephedrine. Norepinephrine and epinephrine drips were started. Also, the FiO2 was increased from 50% to 100%. There was a minimal and transient response to epinephrine administration. The patient was then returned to supine position, and he arrested shortly thereafter. Chest compressions commenced immediately upon loss of cardiac rhythm. The cardiac anesthesia team emergently responded and performed an intraoperative transesophageal echocardiography (TEE), which showed reduced left ventricular ejection fraction and reduced right ventricular systolic function. Due to unsuccessful cardiopulmonary resuscitation, the patient was placed on venoarterial ECMO via right femoral artery and vein; stable hemodynamics were achieved. A total of 8000 units of Heparin was given upon ECMO installation. At this point, the planned surgery was aborted. The patient was transported to the cardiac catheterization lab for pulmonary angiogram, cardiac catheterization, and antegrade perfusion of the right superficial femoral artery. A large thrombus in the left pulmonary artery was discovered on selective angiography (Figures 1–4). Hypothermic protocol was initiated. Heparin therapy was also continued at this point.

On hospital day 5, a CT chest with contrast showed multiple bilateral pulmonary emboli and evidence of right ventricular failure. Right heart catheterization and placement of a Swan-Ganz catheter demonstrated that the patient was found to have severe pulmonary hypertension 55/30 and elevated central venous pressure (CVP) of 18. The patient underwent bilateral pulmonary artery embolectomy, exploration of right atrium with removal of clots, discontinuation of ECMO support, and repair of right femoral artery on hospital day 9. His pulmonary artery pressure and CVP improved to 31/12 and 8, respectively. One month later, the patient was discharged to a rehabilitation facility with a plan for conservative management of his fracture.

## 3. Discussion

Early detection and treatment of PE are essential to improving morbidities and mortalities of patients with traumatic injuries. PE is often diagnosed clinically using the history, vital signs, and symptoms to guide in the detection of a thrombus [5]. PE is often diagnosed clinically using the history, vital signs, and symptoms to guide in the detection of a thrombus. When using pulse oximetry as an indicator of PE, the finding is usually a sudden and drastic drop in oxygen saturation. Retrospectively, the patient's low preoperative oxygen saturation may be secondary to the thrombus in his pulmonary artery (Figures 1–4). Indeed, the development of venous thromboembolism (VTE) likely occurred prior to surgery. He may have had small microemboli in place causing his low oxygen saturation before surgery.

As mentioned earlier, the development of venous thromboembolism (VTE) likely occurred prior to surgery. Major trauma often leads to the risk factors in Virchow's triad or hypercoagulability, endothelial injury, and venous stasis. The patient might have had microembolies derived from peripheral bone marrow cellular aggregates trapped in the lung vessels, causing his low oxygen saturation before surgery. Moreover, his injury caused direct disruption to the endothelial glycocalyx layer (EGL), which leads to release of both procoagulant and anticoagulant factors though procoagulant ones prevail [6]. This endothelial activation after trauma may be caused by vasoactive catecholamines, inflammatory mediators such as tumor necrosis factor-alpha (TN F-*α*), thrombin, and hypoxia [7]. This can lead both to pulmonary microemboli as well as the formation of larger deep venous emboli.

Immobility and reduced blood flow from the injury also contributed significantly to VTE development in this patient. On a microscopic level, hypoperfusion is associated with decreased level of protein C, which is an important anticoagulant because activated protein C deactivates factor Va and VIIIa [6]. Activated protein C mediated fibrinolysis is hindered as well. Trauma induced coagulopathy is a complex process, and both microembolism and classical pulmonary embolism derived from a peripheral DVT were at play in this case – leading both to preoperative mild hypoxia events, and an acute catastrophic event on positioning. The inciting event causing a venous thrombus to detach and embolize is often unknown [8], but can be associated with clot propagating maneuvers, as there have been case reports citing tourniquet placement as the initiator of clot migration [5]. Subsequent repositioning of our patient in the operating room may have caused a larger venous thrombus to become dislodged and embolize to the pulmonary arteries, leading to cardiac arrest.

Pulmonary angiogram is the gold standard for diagnosis, but it is often possible to begin the evaluation with a less invasive test. Intraoperative TEE is extremely useful for monitoring and diagnosis. One study discovered that in 19 out of 22 cardiac arrests, TEE was successful in establishing a diagnosis [9]. In addition, TEE provides a survival benefit, allowing clot visualization and initiation of specific treatment plans [2, 9]. Orthopedic and trauma patients are some of those at highest risk for thrombi, but cardiac anesthesiologists are seldom found administering these anesthetics. Although right ventricular strain is the most common finding in these cases, our patient showed a global deterioration [9]. One explanation is that the patient's extensive fracture resulted in occult bleeding which contributed to severe hemodynamic instability and cardiac arrest.

ECMO has been previously described as a treatment modality for patients with massive pulmonary embolism and resulting shock [4, 10, 11], but it is not without significant risk. Dolmatova et al. described five cases of near fatal pulmonary embolism in which ECMO was used. In these cases the overall mortality was 40%, with one death resulting from an ECMO-related complication and another death from the inability to maintain cerebral perfusion [4]. On the other hand, ECMO has been successfully implemented in patients with pulmonary embolism that remain unstable despite aggressive resuscitation. The 90-day-survival was 47% in one study where ECMO was used in 17 unstable patients with pulmonary embolism [11]. In the same study, fifteen (88%) patients suffered severe hemorrhage, but there was no influence on overall survival [11]. In a review of case reports and case series published over the past 20 years, there was an overall survival rate of 70% in patients with massive PE. When comparing thrombolysis, catheter embolectomy, and surgical embolectomy, the mortality was not affected by the treatment modality. However, patients who had ECMO instituted during cardiorespiratory arrest had a higher risk of death [5].

Trauma patients are at increased risk of VTE due to the presence of Virchow's triad of hypercoagulability, endothelial injury, and venous stasis [1]. This patient likely experienced all three. Injury to blood vessels can cause intimal damage that results in thrombosis. Prolonged bed rest and hypoperfusion cause venous stasis. A hypercoagulable state results from decreased levels of antithrombin III and suppression of thrombolysis [1]. Because of this patient's extensive fracture, his risk of VTE was particularly high. The benefits of starting anticoagulation early may outweigh the bleeding risks of doing so prior to surgery. Looking back at the course of this patient, the time from injury to repair was prolonged by interhospital transfer and initial attempt to perform closed reduction of his fracture. During this two-day period, the patient may benefit from multiple doses of anticoagulation with close monitoring for bleeding (hemoglobin and hematocrit, imaging) with the intention of holding anticoagulation just prior to the operation. However, frequently studies focus on prevention of VTE events after orthopedic surgeries, and not much has been established regarding the benefits and risks of presurgery thromboprophylaxis regimens [12–14]. Furthermore, most controlled trials compare different anticoagulant medications rather than the preoperative versus postoperative timing of the anticoagulation. In Europe, low molecular weight heparin (LMWH) is traditionally started before surgery, whereas in North America a higher dose of LMWH is usually started postoperatively due to concern for hemorrhage [15]. However, one study compared preoperative and postoperative thromboprophylaxis in patients with femoral neck fractures. They examined 25,019 patients from the Norwegian Hip Fractures Resister who underwent hemiarthroplasties for femoral neck fractures. 99% of these patients received LMWH. They found that starting anticoagulation postoperatively resulted in an increased mortality (RR 1.13) and a higher risk of reoperation (RR 1.19) compared to patients who started anticoagulation preoperatively [15]. Furthermore, there was no difference in bleeding complications. Using a lower dose of LMWH was also associated with the lower mortality and reoperation risk [15]. This study, although not a randomized controlled trial, does support the use of a lower dose of LMWH preoperatively.

The American College of Chest Physicians (ACCP) guidelines recommends the use of low molecular weight heparin for major trauma patients as soon as it is safe to do so [1]. Trauma patients have a high incidence of VTE [16, 17]. However, patient mortality due to PE following total joint replacement was not significantly affected by the type of thromboprophylaxis regimen [14]. After elective total joint replacement in 4253 patients, the incidence of fatal PE was very low (0.07%) [15]. Overall mortality was higher in patients on potent anticoagulants than on patients receiving aspirin combined with regional anesthesia. The incidence of nonfatal PE was also higher in patients on potent anticoagulants. Thus, PE occurs despite the use of anticoagulants [16]. However, these types of elective orthopedic surgeries cannot be directly compared to trauma patients with extensive orthopedic injuries. In trauma patients, the initiation of anticoagulation is often delayed due to concerns of injury associated bleeding. In a multicenter prospective cohort study [16], VTE prophylaxis was initiated within 48 hours of injury in 25% of patients, but 25% did not receive anticoagulation for at least seven days. Early prophylaxis was associated with a 5% risk of VTE. Delay of anticoagulation beyond 4 days resulted in a threefold increase in the risk of VTE. Factors associated with the late initiation of prophylaxis included severe head injury, absence of comorbidities, and massive transfusion [16].

## 4. Conclusion

The current practice of withholding anticoagulation prior to surgery in trauma patients with orthopedic injuries at high risk of VTE is not indicated. The risk/benefit ratio of preoperative anticoagulation must be carefully considered and weighed against the risk of VTE. Further research is needed to clarify the use of preoperative anticoagulation in orthopedic trauma patients.

## Figures and Tables

**Figure 1:** Before injection with catheter in pulmonary artery.

**Figure 2:** Start of injection with contrast showing mainly in the right lung with some contrast in the left upper lobe.

**Figure 3:** After injection with minimal perfusion of the left upper lobe and almost no perfusion of the left lower lobe.

**Figure 4:** After injection without any significant perfusion of the left lung, especially in the lower lobe.
